# Competencies Required to Deliver a Primary Healthcare Approach in the Occupational Therapy: A South African Perspective

**DOI:** 10.1155/2023/4965740

**Published:** 2023-04-13

**Authors:** Deshini Naidoo, Jacqueline Marina Van Wyk

**Affiliations:** ^1^Discipline of Occupational Therapy, School of Health Sciences, College of Health Sciences, University of KwaZulu-Natal, South Africa; ^2^School of Clinical Medicine, College of Health Sciences, University of KwaZulu-Natal, South Africa

## Abstract

**Introduction:**

The South African government introduced a reengineered primary healthcare approach to promote universal health coverage. The approach was to ensure equitable, efficient, and quality health services for consumers in private and public healthcare sectors. The transition toward a more comprehensive primary healthcare approach to intervention requires occupational therapists who predominantly worked in private and hospital settings to extend their services to clients who previously would have had little access to such services. This study was conducted to identify the key competencies required by occupational therapists to deliver appropriate primary healthcare services to communities from previously disadvantaged periurban and rural areas.

**Methods:**

An exploratory, qualitative study design was used. Through the use of policy documents and data from key informants (*n* = 5), established therapists (*n* = 14), and novice occupational therapy graduates (*n* = 39), the study identified and mapped the stakeholders' perspectives of the competencies required by graduates to practice in periurban and rural settings in KwaZulu-Natal in South Africa. Data was collected using semistructured interviews, a focus group discussion, a document review of the university's curriculum, and the local and global regulatory documents. A framework based on the seven roles of the university's competency framework informed the data analysis process. The seven roles are health practitioner, communicator, collaborator, health advocate, leader and management, scholar, and professional. *Findings*. Participants highlighted the need for graduates to have adequate knowledge and understanding of the impact of the Department of Health policies and social determinants of health on occupation and the client's health. They also needed to be suitably skilled in culturally sensitive communication, negotiating shared goals with the stakeholders, and managing a department. Graduates needed to be socially accountable and develop services to advocate for their clients.

**Conclusion:**

The study offered insights into the essential graduate competencies identified by the stakeholders and recommended measures to prepare rehabilitation graduates for service deliver*y* in primary healthcare contexts.

## 1. Introduction

The COVID-19 pandemic has highlighted the shortage of healthcare providers on a global scale. It accentuated the continued inequities to health services for underserved rural and marginalized communities in low- and middle-income countries. The trend to deliver contextually relevant community-responsive health practitioners to serve in the 21^st^ century has been highlighted in the Lancet report [1]. The report recommends that health profession education institutions globally use an interprofessional education approach and ensure opportunities for transformative learning experiences during health profession training. Failure to expose graduates to varied contexts and setting with different socioeconomic determinants of health, cultures, and communities, training in disciplinary silos, and lack of integrative learning experiences are reasons listed in the report as to why graduates are poorly prepared for team-based care and unable to advocate for those in their care. Many countries in the global north and south have since implemented more population- and primary healthcare-based training programmes to address local health and social issues, including facilitating livelihoods and work opportunities through an occupational justice framework [2, 3]. Higher education institutions are therefore urged to expand the use of more innovative, student-centred, and community-engaged health profession education programmes to include training in low-resourced peripheral facilities. Such a shift is believed to promote the development of contextually relevant and work-ready graduates who would be more competent and confident to function in unfamiliar settings and better advocates for the social and health needs of people living in all settings including disadvantaged communities.

The need to increase access to health is central to uplifting people who live in marginalized communities [4]. This need is equally apparent in the South African (SA) society, where access to equitable health care, a constitutional right, remains fragile due to gross neglect during SA's apartheid era. Access to health care in SA predominantly favoured some communities based on ethnicity and geographic locations ([5] : 165). South Africa has since formulated a National Development Plan to address widespread inequality and inequity, including implementing a national health insurance and primary healthcare (PHC) strategy to achieve equitable health for all SA citizens.

A PHC approach is internationally recognised as encompassing the use of a comprehensive promotive, protective, preventive, curative, rehabilitative, and palliative care strategy to prioritize healthcare services for individuals, families, and communities to optimize health and advocate for policies that promote and protect health and well-being [6]. It is envisioned that the integrated health service framework will address individualized health needs through primary healthcare and that the needs of the population will be met through public health functions [6]. The National Health Insurance (NHI) White Paper, which guides public sector service delivery in SA, similarly emphasizes a shift toward a more population-orientated primary healthcare approach to health and well-being [7]. The policy formation has accelerated the need for occupational therapists to embrace more primary healthcare approaches as part of the government's strategy to ensure universal access to healthcare.

In the medical education context, authors have affirmed the role of higher education institutions (HEIs) in ensuring that a socially just approach is followed in activities relating to education, research, and community service to address the priority health needs of local communities [8]. In 2018, South Africa recorded a ratio of 0.9 occupational therapists per 10000 population. Although the number of occupational therapists registered with the Health Professions Council of South Africa has increased to 5638 in 2020 [9], the number is still inadequate to provide for the rehabilitation needs of the population. SA have traditionally trained limited numbers of occupational therapists, which resulted in their preference to working mainly in urban hospital settings and focusing on remedial and rehabilitative interventions at an individual level [10]. After completing a four-year undergraduate degree, occupational therapy graduates are regarded as qualified to enter public practice in the SA setting. New occupational therapists have experienced difficulty in delivering PHC services due to their lack of preparedness to cope with cultural differences and inadequate exposure to the needs of people living in periurban and rural communities during their training period [10, 11].

From a global perspective, Dahl-Popolizio et al.'s [12] commentary proposes that occupational therapists can assist in health promotion and disease prevention and reduce the development of chronic and noncommunicable diseases by working with clients and communities in primary healthcare settings. Occupational therapists' unique approach of addressing the whole person offers an opportunity to address health behaviours by considering strategies that address the client's context, value system, habits, community, and culture. Other researchers including Halle et al. [13] and Wood et al. [14] also highlighted the value and role of occupational therapy in primary care, interprofessional and team-based approaches, and current educational preparation for entry-level occupational therapists and occupational therapy assistants. Similarly, Wilcock and Hocking [15] and Hammell [2] emphasized the unique role that occupational therapists can play as part of an integrated primary healthcare team. Not only can they improve health outcomes by addressing the social determinants of health but they can also work across the lifespan and use a community-/population-based approach to health, health promotion, disease prevention, and lifestyle interventions [14–17]. The shift to integrate occupational therapists into PHC teams in the healthcare context is not unique. Reports have documented efforts to integrate occupational therapists into interprofessional teams in PHC settings in Australia, United Kingdom, and Canada [14, 15, 17–19]. However, there is limited published literature on the competencies required by entry-level occupational therapists for primary healthcare service delivery in African and South African settings.

While South African studies highlighted a need for occupational therapists to work at primary healthcare levels [20, 21], they also acknowledge how human resource constraints led to a prioritization of hospital-based interventions over population-based approaches. In alignment with the White Paper, the Occupational Therapy Association of South Africa (OTASA) formulated a position statement on the proposed roles of an occupational therapist in primary healthcare [22]. The statement emphasizes the relevance of the PHC approach in the South African context, and it supports the inclusion of occupational therapy services in emergent practice settings. The position paper proposes for occupational therapists to play multiple roles at the PHC level. Occupational therapists are expected to accept nontraditional roles in new complex environments, initiate and participate in intersectoral collaboration, and contribute to management structures in the PHC system [16, 19, 21, 22]. For example, in 2019, South Africa, a low-middle-income country, reported a 40.7% unemployment rate amongst 15- to 34-year-olds [23]. This statistic emphasizes the need for occupational therapists to work in PHC settings to provide greater vocational rehabilitation and engage the youth in entrepreneurship.

The position paper further envisaged the need to equip occupational graduates with knowledge, skills, and attitudes for professional practice during their undergraduate education. The vision to ensure that graduates are effectively and authentically prepared to meet service delivery needs in the community and PHC settings saw the implementation of the new vision for occupational therapy education at the local training institution. The shift encompassed clinical rotations for undergraduate students in more authentic community-based and rural training settings. The new training exposures are further from previous hospital-based service-learning sites and encompass a greater primary healthcare focus. [24, 25].

Occupational therapy educators have sought suitable models to express the roles required of competent “ready-to-practice” occupational therapy graduates in the SA healthcare setting. Faculties of health science associated with two South African universities have adopted and implemented a competency framework to inform curriculum design and to ensure that graduates attain the desired competencies as health professionals [26, 27]. This framework, adapted from the Physician competency framework [28], proposes that all cadres of health professionals develop and acquire the necessary skills in seven critical roles before graduation. These graduate competencies include the roles of the health practitioner expert, professional, communicator, collaborator, leader/manager, scholar, and health advocate.

The role of a health practitioner is essential to practice as a therapist. The professional role entails adhering to ethical standards and a commitment to pursue continued professional education. In terms of occupational therapy, graduates must demonstrate the ability to assess the impact of various health conditions on the client's participation in life occupations, advise them on lifestyle modifications to address health risks, and advocate for health and well-being.

Much uncertainty remains over the competency mix required of occupational therapy graduates to meet workplace expectations in PHC settings especially given their new contribution to the healthcare teams in the rural and periurban SA contexts. A preliminary study reported on the challenges experienced by newly qualified graduates working in PHC in periurban and rural settings [10]. These challenges include a vague understanding of the PHC approach and being unaware of the realities of practising in a rural resource-constrained environment. They also lacked exposure to primary healthcare clinics during their training.

Despite the adoption of a generic competency framework to inform the education and training of all health profession students by the institution, an effective curriculum response for occupational therapy service in the KZN context requires a needs assessment to improve the alignment of curriculum goals, learning objectives, and clinical exposures to produce a “fit-for-purpose” and ready-to-practice occupational therapist. The South African health system is regulated at a national and provincial/state level. The occupational therapy programme at our institution is closely aligned with the KwaZulu-Natal Department of Health (KZN-DoH) which is the provincial government authority. KZN-DoH has mandated that health science programmes produce graduates who are capable of delivering services appropriate for periurban and rural hospitals in KZN.

This study was conducted as part of the curriculum review process [29] at one South African Higher Education Institution. The objective was to identify and report on the views of multiple stakeholders (including global and national accreditation guidelines) to define the competencies required by an occupational therapist to function at a primary healthcare level in the KwaZulu-Natal context.

## 2. Methodology

### 2.1. Study Location and Context

The study was conducted at a South African university that offers occupational therapy education in the province of KwaZulu-Natal. The occupational therapy programme is a four-year entry-grade undergraduate programme. The curriculum comprises four main pillars: occupational therapy theoretical constructs and ethical practice, occupational therapy professional practice, research, and service-learning rotations. Students deliver services during four-six to eight-week rotations in their final year in an acute hospital or nongovernmental organizational setting. One of the rotations occurs in a community setting where the students work as part of a multidisciplinary team and engage with community stakeholders.

KwaZulu-Natal is one of the more densely populated provinces with a mix of urban, periurban, and rural populations. It has the second-highest population in South Africa. It has a high disease burden, including decreased maternal, newborn, and child health; HIV and TB; noncommunicable diseases such as hypertension, diabetes, and stroke; and a high level of violence and injuries due to trauma.

### 2.2. Research Orientation and Design

This study was conducted to gain insight into the competencies required by occupational therapy graduates to serve in primary healthcare practice. An interpretivist paradigm guided the qualitative study. Data collection included focus group discussions, semistructured interviews, and the analysis of policy and training documents. The interpretivist paradigm recognizes “knowledge” as being socially constructed through the subjective views of the participants [30]. The subjectivist epistemological position was assumed in that the participants and the researcher coconstructed the data during the interviewing process. This position acknowledges the specific beliefs of participants about their realities and life experiences within a specific social context. The interpretivist paradigm allowed for the exploration and insight into multiple and possible diverse interpretations of reality rather than seeking a “single truth” for the data [30].

A purposive sampling strategy was used to invite representatives who are most knowledgeable and engaged with graduates from the occupational therapy programme. This strategy allowed for exploring multiple participant perspectives and acknowledging each participating group's perspective as being embedded within the setting, culture, and unique life experiences. The three participant groups that were recruited included stakeholders from the KwaZulu-Natal Department of Health (KZN-DoH). As employers, they work closely and manage entry-level, novice, and established occupational therapists. Five key KZN-DoH participants (*n* = 5) represented the management group. These key informants served as managers in PHC and rehabilitation at a national, provincial, and district healthcare level (see Table 1 for inclusion criteria).

Fourteen established occupational therapists were invited, and thirty-nine novice occupational therapists who worked in periurban and rural areas were recruited from the higher education occupational therapy 2012, 2013, and 2014 graduate cohorts (see Table 1 for inclusion criteria). Established occupational therapists are defined as those who had had been working for more than four years in a public sector hospital or at nongovernmental organizations in one of the two KwaZulu-Natal geographical districts where students are placed.

All participants were recruited via email or telephonic communication. Information relating to the study and an informed consent document were sent to those interested in participating before the interviews.

The perspectives of novice and established practitioners assisted in gaining an understanding of the competencies required from both perspectives as these participants had experience working in PHC settings in KZN and had been exposed to the occupational therapy curriculum at the higher education institution. The selection of these participants assisted in obtaining perspectives that were rooted within the participants' experiences of working or living within the South African context and contributed their specific experientially based perceptions of delivering a PHC service from a grassroots worker level to that of a national manager level.

### 2.3. Data Collection

Data was collected using semistructured interviews and focus group discussions with the key informants from the KZN-DoH, established occupational therapy practitioners, and novice service occupational therapists (see Table 1) by the primary author. The primary author is a university academic with experience in qualitative data collection methods. The core question that guided the interviews was “What competencies are required by a new occupational therapy graduate to deliver a service in the PHC setting?” The focus group was held in person at a venue and time convenient to the participants. The focus group was conducted in English for approximately 90 minutes. The focus group allowed the participants to share their views in a supportive environment and deepened the discussion. Only one focus group discussion was held due to the availability of participants. The focus group was held after the semistructured interviews. The primary author initially conducted semistructured interviews on a one-to-one basis as this was found to be preferable in terms of convenience for the participants. The participants were given pseudonyms during the semistructured interviews and the focus group discussion. Additionally, a review of relevant documents was conducted using the university's competency framework roles as the lens to explore the global and national training standards and outcomes and the university's perspectives on the competencies required for practice (Table 1).

### 2.4. Data Analysis

A hybrid approach to data analysis as per the protocol outlined by Fereday and Muir-Cochrane [31] was used for data analysis. This process involved both inductive thematic analysis and the use of a deductive a priori template of codes that was based on the competency framework as used at the institution. The codes in the codebook were based on the different roles outlined in the competency framework. After data saturation was reached, the verbatim transcripts from the interviews and focus group were initially read and reread to become familiar with the data. The second reading helped to identify emerging codes. The primary author then applied a template approach. This involved developing a template from codes from a codebook. The codes from the codebook guided in identifying the data sets and organising the text and collapsing the data into themes based on the competency roles. The primary author discussed and verified the codes and the themes with the second author to reach a consensus on the codes and themes and to ensure there was no bias. The second author is a senior researcher with experience in qualitative data analysis. The data review revealed that the participants had only identified five of the seven a priori roles outlined in the codebook. Hence, only five roles are described in the study, namely, health professional, communicator, health advocate, leader/manager, and collaborator. After the roles emerged, the data were categorized into knowledge, skills, and attitudes to identify competencies required by entry-to-practice level occupational therapists. A peer debriefing process with the second author (an educationalist and not a teacher on the programme) allowed us to reach a consensus on the data analysis and extraction process. The authors were aware of their position within the research process. They occupied an insider perspective as all authors were involved in the research and had exposure to the institutional occupational therapy programme.

### 2.5. Ethical Consideration and Trustworthiness

Ethical approval for the study was granted by the Biomedical Research Ethics Committee of the University of KwaZulu-Natal (UKZN-BE248/14) and the KwaZulu-Natal Provincial Ethics Committee of the Department of Health. Principles of confidentiality and the right to withdraw were adhered to in the study. All participants received written and oral information relating to the study before signing the consent forms. Pseudonyms were used to protect their anonymity.

Trustworthiness was operationalized through the triangulation of data to ensure multiple perspectives of the KZN-DoH stakeholders and the occupational therapy stakeholders. Data method triangulation was achieved by using focus groups, semistructured interviews, and document analysis. Member checking was completed at the end of each interview, key points generated through the focus group discussions were summarised, and participants were asked to verify the accuracy thereof. These strategies ensured the credibility of the data. The dependability of the data was achieved through the use of an audit trail. The researcher kept field notes and wrote memos during the data collection and analysis to provide an accurate record of decisions.

## 3. Findings

Participants identified only five of the seven UKZN competency roles as essential for PHC practice. These roles included those of the health practitioner, communicator, collaborator, leader, and health advocate. The roles have been subdivided into the knowledge, skills, and attitudes required of occupational therapy graduates for PHC practice. A summary of the key competencies highlighted by participants is provided below. Tables 2–6 provide more details of the identified themes linked to verbatim quotes to substantiate the relevant roles. Participants are named using numbers to ensure anonymity.

### 3.1. Theme One: Role of a Health Practitioner

The occupational therapist's role as a health practitioner was viewed as essential and central for graduates to deliver equitable PHC services. The knowledge required includes a sound understanding of the PHC approach, the roles expected from graduates at different levels of care, and an overall understanding of how the health systems function. Graduates should have insight into governmental procedures particularly to how policies and procedures impact health and service delivery. Additionally, participants emphasized that graduates should know the contextual, structural, and cultural factors that influence community participation in occupation.

Graduates need context-specific skills that are community-focused that acknowledge the cultural context of the community where they work. They also need profession-specific skills to address prevalent conditions and to deliver contextually relevant and culturally specific interventions in the community context.

Numerous attributes were mentioned relating to this role. It was identified that graduates should be problem solvers, “think out of the box,” adaptable, resilient, persevering, resourceful, proactive, and demonstrate social accountability and empathy. Additionally, graduates need an awareness of the power relationships and to be culturally sensitive when dealing with clients.

### 3.2. Theme Two: Role of a Communicator

Graduates need to be proficient in the local indigenous language and use alternative augmentative communication for communication. Skills required for effective communication include having good verbal and written communication, especially for feedback and for use in managerial positions. Graduates should recognize the political workplace climate and adapt their communication appropriately. If unable to communicate in the indigenous language, the graduate should elicit the assistance of a skilled translator. All participants emphasized the need for graduates to be resilient when receiving feedback and assertive when advocating for change to the health system and to improve population health in community settings.

### 3.3. Theme Three: Role of a Collaborator

Graduates need to demonstrate knowledge and insight into social and health legislation, policy, and procedures to develop and implement collaborative community or multidisciplinary projects. Additionally, participants highlighted the essential need for graduates to understand the benefits of establishing a network. Skills required for collaboration include creating and maintaining a network, collaborating and developing beneficial goals for the client or the project, and working with members of diverse teams. Additionally, graduates should be able to negotiate community entry, demonstrate a willingness to pay attention to stakeholder views, and take cognizance of their concerns.

### 3.4. Theme Four: Role of a Health Advocate

As a health advocate, graduates should know how the health systems interact in the community and how this interrelatedness influences health outcomes for their clients. Furthermore, graduates need insight into their role in empowering the client's ownership of their health and advocating for health promotion. Skills required include serving as an advocate for clients and the community and delivering primary, secondary, and tertiary preventative programmes. They also need to develop partnerships and facilitate task-shifting with community healthcare workers to ensure the continuity of services. The graduates need to demonstrate resilience and persistence to overcome challenges when advocating for clients and programmes.

### 3.5. Theme Five: Role of a Leader and a Manager

Knowledge required for the role of manager and leader includes the ability to evaluate existing services and plan and develop new services as and where required. Graduates need skills to develop policies and procedures, prioritize workloads, and propose changes to improve inefficient systems. Furthermore, graduates need to develop insight into financial management and departmental administration. Being proactive and determined were the attributes highlighted as the most important for the leader and manager role.

## 4. Discussion

The findings from this study provided insight into the essential competencies based on policy directives and stakeholder perceptions as relevant for occupational therapy service delivery at a PHC level. The need for graduates to have expert knowledge and skills was viewed as central in delivering equitable PHC services. The key attributes highlighted include being problem solvers, adaptable, resilient, resourceful, proactive, and empathetic. Participants stressed the need for graduates to be aware of the power relationships and show cultural sensitivity when dealing with clients.

The key considerations for intervention at the PHC level included the consideration of contextual, structural, and cultural factors influencing participation in occupation, social determinants of health, different levels of care, having resource limitations, and implementing health promotion and disease prevention programmes. This finding is aligned with Hammell's recommendation for occupational therapists to actively address the social determinants that obstruct occupational engagement. Such adherence to address the obstacles will promote occupational equity and occupational rights [2]. Additionally, graduates should have an overall understanding of the functioning of the health systems, government processes, and how this potentially influences their occupational therapy practice. The findings of the study concur with the literature on the occupational therapists' role in PHC. [14–17, 19].

The competencies linked to the roles of communicator, collaborator, health advocate, and leader and manager had a greater skill focus. Culturally competent communication was identified as a critical skill to adapt to different political work climates, for networking, and to negotiate community entry and facilitate reciprocal learning in teams. The critical elements for cultural and competent communication in the medical context were previously stressed by Teal and Street [32]. The essential elements in culturally competent communication include recognizing potential differences, incorporating cultural knowledge, and being aware of verbal and nonverbal behaviour when negotiating and collaborating. The literature also reaffirms the need for graduates to use collaborative approaches, to being socially accountable, actively interact with the community, acknowledge their belief systems, and accommodate for perceived power differentials to facilitate productive partnerships with community members [14, 16, 33].

Collaboration, communication, and leadership skills were identified as essential competencies to initiate projects, establish and maintain networks, and facilitate common goals within diverse multidisciplinary teams and with clients, families, and other stakeholders in the community. Skills required for health advocacy included developing primary, secondary, and tertiary prevention programmes, using their understanding of the impact of the health system on the client and communicating to develop health promotion programmes such as early stimulation programmes for children and being able to task-shift to community healthcare workers to ensure continuity of care. Wilcock and Hocking [15] similarly highlighted the need to develop programmes that promote health in the community and focus on illness prevention, chronic disease management, and reduce health risk behaviour. Being a health advocate required graduates to speak up for the rights of their clients—both in the hospital and in community settings. This competency is closely linked to the graduate's ability to recognize social injustice and their knowledge of how to apply policies to consult when advocating for clients and at-risk populations. Similar to the findings in this study, both Wilcock and Hocking [15] and Galheigo [34] suggested that a combination of advocacy, collaboration, and leadership skills should be developed in graduates to allow them to establish programmes and promote for the rights of their clients.

The competencies identified in this study are relevant to both general occupational therapy practice and its practice in PHC settings. It is noteworthy to mention that the stakeholders were uncertain about the role of occupational therapists in the PHC setting. Occupational therapists expressed limited views on the competencies required by graduates to practice health promotion and prevention in PHC settings which may be due to their lack of training and practice experiences in the PHC setting. The uncertainty remains despite the policy imperatives both by SA's National Department of Health [7] and the Occupational Therapy Association of South Africa advocating for more health promotion and prevention in service delivery by public sector therapists [22].

There is thus a need to guard against occupational therapy services slipping back into conventional practices. Braveman [18] suggests that uncertainty about roles and contributions could be due to the occupational therapists' lacking clarity and insight into their roles in the new context and thus being inadequately receptive to potential areas of contribution, which in turn reflects their education and practice exposures during their undergraduate curriculum. Naidoo et al. [21] similarly found that community stakeholders articulated the need for services at a primary healthcare level; however, they were not as vocal on services required for health promotion, consultation roles, and disease prevention.

The competencies identified in this study can inform curriculum development and review to align teaching, learning, and assessment practices with PHC approaches which are now more strongly present in occupational therapy training. Occupational therapy students currently engage with PHC concepts relating to service delivery during a community rotation in their final year. However, a previous study exploring a graduates' ability to implement primary healthcare approaches revealed perceived inabilities to manage cultural differences, to complete administrative and management tasks, and inadequate exposure to the needs of people living in periurban and rural community settings [21].

A possible solution to promote the understanding of the occupational therapy role in PHC and the required competencies needed for successful functioning is to ensure that they are embedded as learning outcomes for students to achieve during their service-learning rotation. It would be essential to inform students of the required competencies that need to be achieved for the successful completion of the rotation. There should be more opportunities for students to practice collaborative goal setting within the multidisciplinary team, intersectoral collaboration with the stakeholders from various government departments in the community, and opportunities to develop and implement health promotion and disease prevention programmes. Students should be expected to implement programmes that promote social justice during service learning in community settings [2].

## 5. Implications for Practice

Occupational therapy educational programmes should produce ethical and socially responsible graduates with the vision, knowledge, skill, and willingness to deliver services to previously marginalized communities.

Educational programmes need to shift their vision and focus from delivering services on a micro- and macrolevel with individual clients in hospital/clinic settings to promoting wellness and population health in community settings.

The critical task for curriculum designers is to consider the needs of the stakeholders during the curriculum review phases to include opportunities to develop, model explicitly, and assess graduate outcomes for PHC settings.

It is hoped that the findings from this study will inform aspects of future training in SA to ensure that graduates are adequately prepared to work in PHC settings. We are acutely aware of the curriculum overload in existing occupational therapy training programmes and how the implementation of these guidelines will require further negotiation amongst curriculum designers.

It should be noted that the findings are generated from a single-site study; therefore, the findings apply to KwaZulu-Natal and are not generalizable. Educators at other higher education institutions would need to review the findings against their specific contexts. It would have been beneficial to include the educator perspective to allow for greater insight and application to the curriculum, but we are confident that this phase generated sufficient insight to continue the ongoing revisions as required on this programme.

## 6. Conclusion

The transition toward a more comprehensive primary healthcare approach to intervention requires occupational therapists who predominantly worked in private and hospital settings to provide a broader scope of services to clients who previously had little access to such services. This study identified critical competencies required of occupational therapists to deliver appropriate primary healthcare services to clients in periurban and rural areas. The findings can inform curriculum review since stakeholders from various sectors identified the essential graduate competencies. The recommended measures also have implications for service training placements to prepare graduates more appropriately for primary healthcare service delivery.

## Figures and Tables

**Table 1:** Data collection methods, participants, and documents used.

Participant group	Data collection method
Key informants from the KZN-DoH (*n* = 5) Inclusion criteria: (i) Managers involved in PHC and rehabilitation who served at a national, provincial, and district healthcare level (ii) Worked in the position for more than two years	Five individual semistructured interviews of 45-60 minutes were conducted face-to-face or via telephone. Interviews were audio-recorded.

Established occupational therapists (*n* = 14) Inclusion criteria: (i) Working more than four years in a public sector hospital or at nongovernmental organizations in one of the two KwaZulu-Natal geographical districts (ii) Established occupational therapists were seen as having the ability to use quick, intuitive thinking to develop goals based on patients' needs and adapt to unfamiliar and unexpected circumstances	Fourteen individual semistructured interviews of 45-60-minute duration conducted via telephone. Interviews were audio-recorded.

Novice occupational therapists (*n* = 39) Inclusion criteria: (i) Worked in periurban and rural geographical areas during their first year of work (ii) Graduated from the education institutions' occupational therapy 2012, 2013, and 2014 graduate cohort (iii) Novice occupational therapists were defined as still dependent on theory and needing to adhere to prescribed protocols and guidelines to deliver services	One focus group with 10 participants. Twenty-nine individual semistructured interviews of 45-60-minute duration, conducted face-to-face or via telephone. Interviews and the focus group were audio-recorded.

Documents	WFOT minimum standards of training (2015) Professional Board for Occupational Therapy, Medical Orthotics and Arts Therapy, Submission for qualification for registration with SAQA (2006) HPCSA Minimum Standards of Training for Occupational Therapy (2009) HPCSA Standards of Practice (2006) University's core competencies for undergraduate students in the College of Health Sciences (2014) All documents were hard copies. University occupational therapy curriculum

**Table 2:** Theme 1: role of a health practitioner.

Description of the theme: This role describes the professional knowledge, clinical skills, and professional attitudes required by occupational therapists for service in PHC settings.

Knowledge: Participants agreed that graduates should plan and implement interventions in resource-constrained settings to address the common conditions in PHC centres. KZN-DoH participants expected for interventions to have a preventative and promotive focus instead of the previous bias toward curative intervention programmes. Furthermore, KZN-DoH and established occupational therapists expressed that graduates should be able to plan and implement interventions in different practice settings. Occupational therapy graduates need to understand the different roles required of them in each location at the different levels of care within the public sector, e.g., hospital, clinic, under a tree, or at a home visit. Both the established and novice occupational therapists verbalized the need for knowledge on structural and contextual factors that impact participation in occupation. Additionally, graduates need to understand the culture of the community that they work in to deliver contextually relevant services. Participants stressed the importance of graduates understanding the impact of health and government policies and procedures on service delivery. The need to understand the effect of health on occupation and its impact on the social determinants of health on the clients' and their families' occupation was highlighted in regulatory documents and emphasized by participants. Novice occupational therapists expressed that graduates should have a firm grounding in the profession. They thought it would help graduates build a solid professional identity, i.e., knowing what OT was and their role in the community, clinic, and hospital. *Apply the occupational therapy process within different fields of practice, with all age groups, and indifferent sectors (health, education, welfare, labour and both in the public and private sectors) describing how the role “fits” and is shaped by the context.* (SAQA exit level outcomes, P4) *For me, they need to know what type of community is that, what belief systems are there or how do you integrate your western type of knowledge within the community knowledge that is already there but how do you use the skills, the profession in a way that will be integrated into the knowledge that is already existing in that particular community, for me that's Number 1.* (Participant 24, novice occupational therapist) *I think you need to really understand the framework that you fitting into, that you being plugged into. I knew public health, I knew how governments sort of worked but I did not understand the context fully, I did not know, not the chain of command but there's certain ways that things happen in government and you have to understand that.* (Participant 34, novice occupational therapist) *Knowledge about human rights about health and well-being, cultural understandings of health and well-being, social determinants of health and well-being, national health needs, priorities and goals, education and disability systems, and the relevant health, social, disability, and workplace legislation.* (WFOT minimum standards (2015), lines 1211-1215) *They need to know how (the) Department of Health works because everything is politically pre-set. You have to know what the government of agriculture is. Other departments, including (the) municipality, they have a section that addresses disability… they need to know what they do. So that we can network.* (Participant 5, established occupational therapist)

Skills: There was a consensus that graduates should conduct vocational assessments and rehabilitation and establish mental health programmes and group therapy in the community. Novice occupational therapists focused on basic assessment and intervention skills, while the KZN-DoH participants and the established occupational therapists reported that graduates must acquire skills to offer services relating to interventions in the community, e.g., home visits, support groups, and caregiver training. Both the established occupational therapy and KZN-DoH participants expressed the importance of educating communities about child development, stimulation programmes, and establishing programmes to address primary, secondary, and tertiary disease prevention. Both the established occupational therapists and KZN-DoH participants emphasized that graduates had to ensure the continuity of interventions through home programmes and collaborate with community health workers (CHW). All participants expressed that graduates should be skilled in prescribing appropriate wheelchairs, completing administrative procedures to obtain devices, and conducting wheelchair maintenance. Established occupational therapy and KZN-DoH participants agreed that graduates need to be critical in their reflections when assessing the effectiveness of interventions. They are advised to learn from their own experiences and that of their peers. In addition, established occupational therapists indicated that graduates should set goals in partnership with their clients rather than impose their views of therapeutic goals. Finally, both the established and novice occupational therapists stressed the need for graduates to understand their role as brand ambassadors. They thought that being a brand ambassador could be strengthened through successful PHC programmes and consistent intervention services in the hospital and the community. *Need to be community orientated department. So, we do our work in the hospital, but we need to ensure that there's community outreach. And with outreach, we take the service out even to the homesteads [more rural homes]. We visit schools, we visit even the pension pay points at some stage.* (Participant 5, established occupational therapist) *You need basic skills. I think whatever the campus prepares you for assessment treatments…that are basic, you have to have that. I think if you do not come out of campus knowing your basic skills, then you are in trouble.* (Participant 28, novice occupational therapist) *Then skills, obviously basic splinting skills, basic skills and exposure to making other assistive devices, basic sewing skills for pressure garments, like general rehab skills and vocational assessment and intervention.* (Participant 32, novice occupational therapist) *Being able to offer services and empowerment to the patient in their community so I think primary healthcare must happen in the community, it must happen with the patient, where he can access services right there, it must empower the patient to feel like he's in charge of his health and it must provide knowledge and skills for the person to be able to live healthy lifestyles...so a lot of preventative and promotive activities need to be done in primary healthcare...and screening for existing disability and existing occupational problems so that we can make the community more independent and empower them to be better.* (KZN-DoH national manager)

Attitudes: Both the novice and established occupational therapists and KZN-DoH participants had strong opinions about the softer skills needed to enable holistic practice. They listed attributes, including graduates having to be adaptable, resilient, persevering, resourceful, proactive, and demonstrate social accountability and empathy. Furthermore, graduates should be problem solvers who are able to think “out of the box” and prepared to learn from seniors and peers. Novice occupational therapists believed that graduates should have a strong work ethic, especially in the face of challenges and poor work ethic sometimes displayed by healthcare colleagues. Furthermore, graduates must be educated about cultural awareness and recognize their power positions over their clients, families, and the community. Novice occupational therapists stressed the importance of being passionate about their profession and a willingness to exceed expectations. Finally, novice occupational therapists reported that they viewed established occupational therapists as mentors and accessed them for peer support when faced with challenging situations. *…must be adaptable, resilient persevere, be resourceful, proactive, be able to problem-solve and be willing to learn from senior staff and peers.* (Participant 10, established occupational therapist) *When you are treating the patients themselves, it's also your attitude towards the patients…, if you do not have the right attitude, the patient will not allow you to treat them or touch them. so you always have to be very open and friendly.* (Participant 20, novice occupational therapist) *Independence and confidence in their abilities. And also not to give up so like problem-solving skills, problem-solve and do not give up. Passionate about what they do. Someone willing to go above and beyond for others, especially in OT. It was so easy just to do nothing and just sit in the office all day because we did not get referrals; I did not do that because I am passionate about OT and helping the community.* (Participant 20, novice occupational therapist)

**Table 3:** Theme 2: role as a communicator.

Description of the theme: This role involves the ability to gather information essential for healthcare, to maintain relationships with clients and their caregivers, and to share the information as appropriate.

Knowledge: All participants and the regulatory documents highlighted the need for graduates to have a good understanding of communication. All participants indicated that graduates need to understand the local indigenous language and understand how the language is embedded in cultural practices. Novice occupational therapists emphasized the requirement to be proficient in isiZulu as it is the dominant language of their clients. Thus, the institution should continue to train and assess isiZulu (indigenous language) communication competency during undergraduate training. Both the novice and established occupational therapists reported that graduates should have knowledge about basic alternative augmentative communication options when treating clients with language—or hearing afflictions. *Knowledge and skills to recognise different political climates in the workplace and adapt communication accordingly.* (Kate, established occupational therapist) ……*need to have more isiZulu (indigenous language), if you have a practical exam and you have Zulu patient you should have to speak Zulu to them. You should be assessed on this so that you make sure you learn it.* (Participant 30, novice occupational therapist)

Skill: There was a consensus that graduates must be proficient to give verbal and written feedback to peers. They also need to communicate to managers about their clients, interventions, and services. The established occupational therapists and DoH participants stressed that graduates had to recognize different political climates in the workplace and adapt their communication accordingly. All participants reported that graduates should adjust their communication style to converse with diverse populations. Skills highlighted included communicating in the clients' first language or using a translator to obtain the clients' history, home environment, and systems for support and explain the purpose of therapy. Both the established and novice occupational therapists endorsed the documentary guidelines for graduates to interact and convey knowledge and information in a culturally sensitive way. Furthermore, established occupational therapists and DoH participants emphasized that graduates should be aware of power relationships when communicating with clients, families, CHWs, and the community. Novice occupational therapists expressed that graduates should learn to communicate with difficult clients and staff, e.g., an angry client. *You have to be a good communicator …It was only about a month down the line that I actually started going to speak to people about how things work; I think it would have been better for me to go and introduce myself to the nursing manager and say this is who I am and this is what I do to get people like that on your side at the end of the day.* (Participant 34, novice occupational therapist) *To adapt their communication style to converse with diverse populations and be cognizant of the power differential when communicating with clients, families, community health workers (entry-level health workers) and the community*. (Participant 14, established occupational therapist)

Attitude: Established occupational therapists and DoH participants noted that graduates should be more resilient when receiving critique or feedback from colleagues, management, and clients. In addition, both the novice and established occupational therapists reported that graduates must, where appropriate, should use assertive communication with their team to motivate for changes to improve the functioning of systems in the community or their institutions. *Evaluate yourself when you get feedback and be able to accept criticism, but know that some people cannot criticise constructively,* (KZN-DoH provincial manager) *Use assertive communication with team and clients and be able to motivate for changes to systems…you need to be proactive. For example, I had to negotiate with the nurses and doctors to allow for screening of clients in the clinic, rather than waiting for a direct referral.* (Participant 22, novice occupational therapist) *Address them[clients and Multidisciplinary team] professionally and politely and you will (be) getting your point across because once you start (showing) emotions, it goes out the window and people will close their ears and not listen to you*. (Participant 3, established occupational therapist)

**Table 4:** Theme 3: role as a collaborator.

Description of the theme: This role described the therapists' knowledge, skill, and willingness to work effectively with others, as a team member, in the health system, and with community stakeholders.

Knowledge: There was a consensus that graduates should be knowledgeable about their roles and how to plan holistically with the multidisciplinary team. Additionally, graduates need to know the social and health legislation and procedures as it will help them understand the contextual and structural factors impacting the project development and implementation of programmes. In addition, occupational therapists expressed the need for graduates to build networks with nongovernmental organizations (NGOs) and government departments to deliver social services. *They [graduates] need to know what can I do here [with the patient]. The Physio can do this, but the OT can do this, and the Speech can do this, but we are all three fitting with this patient. We are planning, together, the treatment goal that will take this patient from here and back to the home.* (Participant 3, established occupational therapist) *So coming here [rural hospital], if I say when a tribal authority meets on a Tuesday, I am expecting the graduate to understand community entry and that I would expect them to have the knowledge to say: maybe you take me to introduce me first, then I will run along with it*. (Participant 5, established occupational therapist) *You need to have partnerships with the nurses and other MDT they would be an intricate part of screening for me, you know because I wasn't able to be everywhere at once, so that collaboration was pretty much key to me having a smooth running department*. (Participant 18, novice occupational therapist) *When you enter into a community, you need to understand the system and the structures that are there. For example, if you go into an urban community, you will find civic organisations, municipal counsellors and all that. So, you do need to be able to collaborate with all the stakeholders*. (KZN-DoH national manager) *Engage relevant role-players as partners in the process of restoring occupational justice and occupational balance.* (HPCSA minimum standards of training, P9)

Skills: As indicated in the legislative documents, all participants agreed with the need for graduates to create and maintain networks and work in diverse teams. Both the novice and established occupational therapists thought it essential to work in teams for holistic service delivery and to engage in a multidisciplinary practice. Both the established and novice occupational therapists mentioned that graduates should be resourceful and establish networks in the community for successful project development. There was a consensus that graduates should develop collaboration and negotiation skills to access networks to determine existing programmes and services, e.g., support groups. They also expressed that graduates should learn negotiating skills to deal with developing goals with multidisciplinary team and stakeholders to ensure project goals that are mutually beneficial to the population the project would serve. All participants stressed that graduates should use appropriate approaches to enter the community. They should introduce themselves to recognize community leaders that serve as gatekeepers in the community. *Learning how to negotiate and meet halfway with them [community] to get what you want and let them [community] get what they want; that is a useful skill.* (Participant 32, novice occupational therapy) *They must build networks with non-governmental organisations (NGOs) and other government departments such as the department of social service and DOE*. (Participant 8, established occupational therapist)

Attitudes: Both the novice and established occupational therapists mentioned that graduates should demonstrate a willingness to value the stakeholders' views and consider their concerns. The national and global regulatory documents highlighted a similar attitude. Graduates should develop and maintain trust and mutual respect with professional and nonprofessional staff. Such relationships with role players were deemed essential to forming successful partnerships in the community setting. Novice occupational therapists found that having a volunteering spirit on the stakeholder and NGO projects had helped them to strengthen their working relationships with these groups. *… need trust and mutual respect with both professional and non-professional staff in the hospital, e.g. if you work with maintenance, you can get assistive devices made.* (Participant 35, novice occupational therapist) *The fact is that in any community you have got to listen. They [graduates] need to be humble and listen to what others and the client is saying. I do not think we teach our students enough to listen. We're so busy teaching them how to give answers. We do not have to know the answers. We've just got to know where to get the help.* (Participant 7, established occupational therapist)

**Table 5:** Theme 4: role as a health advocate.

Description of the theme: This role pertains to advocating for the client, the community, and, through preventative and health promotion programmes, to advance services that contribute to positive health outcomes for individuals and members in the community.

Knowledge: DoH participants expressed that graduates had to know and understand how the health system interacted with the clients and the community and how the interrelatedness impacted health outcomes. Novice occupational therapists thought that graduates required knowledge of governmental procedures of the Department of Health and the Department of Education to facilitate the referral of clients. Established occupational therapists mentioned that graduates should know and understand their role in empowering a client to take ownership of their health and in health promotion programmes. *Graduates need to have the knowledge, skill and willingness to conduct interventions in the community and clients” homes*. (Participant 4, established occupational therapist) *They need to have knowledge of what goes on behind the scenes, you can make such a difference to somebody's life if you aren't just focused on treating them. ...like someone who is travelling from really far and has an appointment at your tertiary hospital, go and speak to an operational manager of one of the wards and find out if the person can come in the day before and stay at the ward overnight so that hey not travelling in the dark.* (Participant 18, novice occupational therapist)

Skills: The DoH participants stated that graduates also needed to serve as advocates for those they served, e.g., if the client was paraplegic. Still, roads were not adequate for wheelchairs; the therapist needed to contact other role players such as municipalities or human settlements to facilitate better road conditions. All participants expressed for graduates to acquire skills in delivering primary, secondary, and tertiary prevention programmes. For example, graduates should implement educational sessions to prevent secondary complications, training about income generation, disability awareness, and awareness groups about health risks. The DoH participants stressed that graduates needed to build the capacity of the CHWs through partnering with them in therapy sessions to ensure task-shifting. They would also have to explore new and nontraditional roles such as being a consultant in a health promotion programme rather than offering direct services. *Graduates must be advocates for the clients they serve*. (Participant 24, novice occupational therapist) *I feel like people with disabilities, they [PWD] do not know their rights*… *I think empowerment and education they fall hand-in-hand with what graduates need to be able to do because there is no one else providing them with that information. As a small district hospital, we as a rehab team are often involved in the empowerment and education of the client to be able to advocate for the person with a disability. So I think it is definitely in a rural setting, I think empowerment and education are extremely important.* (Participant 1, established occupational therapist) *... If you have a paraplegic client, but roads are not adequate for wheelchairs, the therapist needs to contact other role players such as a municipality or human settlement to facilitate better road conditions.* (KZN-DoH national manager)

Attitudes: All participants noted that graduates must persevere and negotiate politics in the community and clinical settings despite the obstacles and challenges they would face. *Those politics, you know, being able to be that advocate to make sure that they know that it is needed even if there are challenges*. (Participant 27, novice occupational therapist) *An example of advocacy. My patients travelled a great distance and needed to go to a tertiary hospital using hospital transport. I had to negotiate with the ward for the mother and child to stay the night so that when they [the patients] saw the specialist they would better utilise the consult*. (Participant 35, novice occupational therapist)

**Table 6:** Theme 5: role as a leader and a manager.

Description of the theme: This role describes the knowledge, skills, and attitudes in leadership required for professional practice, managing of a department, and contributing to healthcare service improvements.

Knowledge: All participants articulated that graduates should know how to evaluate existing services and be able to develop new services. The need for graduates to know the budgets and management of a department was highlighted in the national regulatory documents. The DoH participants particularly stressed that graduates should acquire some understanding in financial management and administration to lead a department effectively. *Prepares estimate budgets for management of own department.* (HPCSA standards of practice, P7) *We [established occupational therapists] do a lot of admin which I think they have[graduates] realised, we do a lot of admin and stats, we do a lot of ordering and they do not know how that works but I suppose I'm saying if it's something they could maybe learn...* (Participant 5, established occupational therapist) *I wasn't prepared for anything admin related. I thought I would get instructions from my supervisor, but it did not happen like that.* (Participant 30, novice occupational therapist)

Skills: The DoH stakeholders emphasized the need to develop policies and procedures for the department. Novice occupational therapists verbalized the need to prioritize their workload in balancing administration, hospital patients, and community work. Both the DoH participants and novice occupational therapists agreed that graduates must develop and implement new services after negotiations with the relevant stakeholders or propose changes to inefficient existing services. This was particularly relevant in cases where recent graduates served as the only therapist. However, in the face of resource limitations, established occupational therapists warned that graduates should learn to build on previous successes and evaluate the success of existing services before they attempted to develop new ones. *I can go to my medical manager and say, ‘can we change the admission form a little bit?' but my medical manager will ignore me. So being able to know how to propose changes would be nice,* (Participant 27, novice occupational therapist) *There's your operational plans, there's your national cost standards, there's your statistics for every day and for every week and for every month, there's your ordering of equipment, there's your cash flow; knowing your stuff and how much budget is allocated to you.* (Participant 4, established occupational therapist) *They [OT] need to learn how to develop a new service, how to work in an existing service and how to plan services, what to look out for if you are an occupational therapist.* (KZN-DoH, district manager)

Attitudes: Occupational therapists emphasized that graduates must be proactive and determined to manage leadership tasks. *...You need to be proactive. I had to negotiate with the nurses and doctors to allow for screening of clients in the clinic, rather than waiting for a direct referral*. (Participant 22, novice occupational therapist)

## Data Availability

Data is available on request.
